The article "Growth and tuber yield responses of potato (Solanum tuberosum L.) varieties to seed tuber size in northwest highlands of Ethiopia" was retracted in 2025. Reason: plagiarism.

# Growth and tuber yield responses of potato (*Solanum tuberosum* L.) varieties to seed tuber size in northwest highlands of Ethiopia

**DOI:** 10.1016/j.heliyon.2023.e14586

**Published:** 2023-03-13

**Authors:** Daniel Asnake, Melkamu Alemayehu, Semagn Asredie

**Affiliations:** a Department of Horticulture, College of Agriculture and Environmental Sciences, Bahir Dar University, P.O. Box 5501, Bahir Dar, Ethiopia; b Director, Technology Multiplication Seed Research Directorate, Amhara Agricultural Research Institute, P.O. Box 257, Bahir Dar, Ethiopia

**Keywords:** Belete variety, Gudanie variety, Potato, Seed tuber size, Tuber yield

## Abstract

Field experiment was conducted during the 2019 irrigation season to evaluate the growth and tuber yield responses of potato varieties in the highlands of Ethiopia. The treatments consisted of four potato varieties (Belete, Shonkolla, Gudanie and Local) and three seed tuber sizes (small (31.5 ± 2.5 g), medium (57 ± 2.5 g) and large (77.5 ± 2.5 g). The experiment was laid out in factorial arrangement using randomized complete block design with three replications in factorial arrangement. The results showed that, variety and seed tuber size in their main effects significantly influenced almost all the tested parameters of potato. Tuber size and variety also interact to influence days to 90% maturity, plant height, large-sized tuber yield, marketable and total tuber yields. Large-sized seed tubers of Belete and Gudanie varieties recorded the highest marketable tuber yields of 39.13 t ha^−1^ and 38.63 t ha^−1^, respectively while the lowest (12.12 t h^−1^) was recorded from local variety planted using small-sized seed tubers. Large-sized seed tubers of Gudanie variety gave the highest net benefit (131,376.50 ETB ha^−1^) with unacceptable marginal rate of return (<100%) while Belete variety with small-sized seed tubers recorded the highest marginal rate of return (1657.14%) with relatively lower net benefit. Optimizing the seed tuber size is therefore necessary to increase productivity and profitability of potato production. In this regard, Gudanie variety combined with medium-sized seed tuber recorded relatively higher net benefit (123,410.80 ETB ha^−1^) with acceptable marginal rate of return (100.9%). Accordingly, production of Gudanie variety using medium-sized seed tubers (57 ± 2.5 g) could be recommended for the economical production of potato and improvement of the income and food security of the smallholder farmers in the study area and areas with similar agro-ecologies.

## 1 Introduction

Potato (*Solanum tuberosum* L.) is one of the most productive food crops in terms of yield and quality protein per unit area and unit time. It is regarded as a high potential food security crop because of its ability to produce high yield and quality product per unit input with a shorter crop cycle [1]. Potato is one of the major crops produced and consumed in the world [2,3]. World annual production of potato is estimated to 359,071,407 tons, which was produced on 16,494,810 ha of land [4]. Despite the high quantities of potato produced worldwide, there are yield gaps due to challenges including abiotic stresses, pests, climate changes and poor production practices [5]. Bridging the yield gaps in potato will ultimately help to ensure securing current and future food security [3]. In this regard, Devaux et al. [1] reported the positive contribution of potato in alleviating food security problems and improving the incomes of smallholder farmers in developing countries under high population pressure.

The article "Growth and tuber yield responses of potato (Solanum tuberosum L.) varieties to seed tuber size in northwest highlands of Ethiopia" was retracted in 2025. Reason: plagiarism.

About 70% Ethiopian′s arable land is found in highlands of the country, which is suitable for the production of potato [6]. Potato is a staple food and plays a significant role in ensuring food security and livelihood improvement in Ethiopia [7]. However, the productivity of potato (13.3 t ha^−1^) is very low [8] compared to the world average (20.11 t ha^−1^) as well as other African countries like South Africa (37.3 t ha^−1^), Algeria (31.2 t ha^−1^) and Egypt (29.2 t ha^−1^) [4]. Many diverse and complex biotic and abiotic factors are contributing for low productivity of potato including inappropriate agronomic practices, prevalence of disease and insect pests, poor soil fertility management, high cost of seed tubers, inadequate storage and marketing facilities [9].

Using optimum-sized and disease free seed tuber is a prim prerequisite for successful production of potatoes. According to Simon [10] and Zeleke et al. [11] seed tuber size and variety of potatoes significantly influenced the performance of potatoes both in terms of quantity and quality. Large-sized seed tubers of improved varieties generally performed well in terms of tuber yield and quality compared to small-sized seed tubers [10]. Smallholder farmers in Ethiopia however are using seed tubers with wider size ranges (28–55 mm in diameter or 39–75 g in weight) for the production of potato without considering the varieties used and the environmental and edaphic conditions of the production areas [12]. On the other hand, tuber size of potatoes varies with variety and the growing conditions of the given area [13].

The quantity of seed tuber required to cover a given area is relatively high (1.8–2.2 t ha^−1^), which significantly increases the production costs and reduces the profitability of potato production. Optimizing the seed tuber size is therefore necessary to reduce the seeding rate and improve the economical production of potato [13,14]. The present study was therefore initiated with the aim of improving the income and enhancing the food security of smallholder farmers by identifying the optimum seed tuber size for economical production of potato.

The article "Growth and tuber yield responses of potato (Solanum tuberosum L.) varieties to seed tuber size in northwest highlands of Ethiopia" was retracted in 2025. Reason: plagiarism.

## 2 Materials and methods

### 2.1 Description of the study area

The experiment was conducted on farmer′s field in *Sahrina kebele* of Farta District, Northwest Ethiopia during the 2019 irrigation season. The experimental site is located at 11° 48' 370'' N latitude and 038° 07' 402'' E longitude with an elevation of 2790 m above sea level. According to Bahir Dar Meteorology Service Center (unpublished), the area received an annual mean rainfall of 1522.5 mm for the last 10 years (2008–2018). The mean maximum and minimum temperatures of the area were 22.5 and 9.4 °C, respectively.

### 2.2 Description of experimental materials

Improved varieties of potato namely Belete, Shonkolla, Gudanie and local variety (*Key Dinch*) were used as test crops. Belete and Gudanie varieties were released by Holetta Agricultural Research Centre in 2009 and 2006, respectively, while Shonkolla variety was released by Awassa Agricultural Research Center in 2005 [15]. The altitude requirements of Belete, Shonkolla and Gudanie varieties are 1600–2800, 1700–2700 and 1600–280 m.a.s.l, respectively. The rainfall requirements of Belete, Shonkolla and Gudanie varieties are 750–1000, 980–1398 and 750–1000 mm, respectively. Belete, Shonkolla and Gudanie varieties matured in 110, 120 and 120 days, respectively [12].

### 2.3 Treatments and experimental design

The treatments consisted of four varieties of potatoes and three seed tuber sizes (small (31.5 ± 2.5 g), medium (57 ± 2.5 g) and large (77.5 ± 2.5 g). Seed tubers were categorized based on Lung’aho et al. [16]. Seed tubers used in each category in the present study were uniform in weight where the maximum weight difference between the seed tubers in a given category was about ±2.5 g.

The treatments were laid down in Randomized Complete Block Design (RCBD) in a factorial arrangement with three replications. Each plot has 3.75 m width and 3 m length with gross and net plot areas of 11.25 m^2^ and 5.4 m^2^, respectively. The distances between plots and blocks were 0.5 and 1 m, respectively. About 50 plants at the spacing of 0.75 and 0.30 m between rows and plants, respectively, were planted in each plot as recommended by EIAR [17].

### 2.4 Management of experimental plants

The experimental land was ploughed using oxen to a depth of 25–30 cm and experimental plots were prepared based on the pre-determined design. Healthy and well sprouted small (31.5 ± 2.5 g), medium (57 ± 2.5 g) and large (77.5 ± 2.5 g) sized seed tubers of each variety were planted. Experimental plots were fertilized with NPS and urea at the rates of 180 and 176 kg ha^−1^, respectively [15]. All other management practices such as weeding, hoeing, earthing-up, pest control were done uniformly for all plots [17].

The article "Growth and tuber yield responses of potato (Solanum tuberosum L.) varieties to seed tuber size in northwest highlands of Ethiopia" was retracted in 2025. Reason: plagiarism.

### 2.5 Data collection

#### 2.5.1 Phenological parameters

Days to 50% emergence was recorded by counting the number of days elapsed from planting up to the date when 50% of planted tubers in the plot were emerged. Similarly, days to 50% flowering was recorded by counting the number of days elapsed from planting up to the date when 50% of the plants in each plot has started flowering. Days to 90% maturity was recorded by counting the number of days from planting up to the date when 90% of the plants in each plot showed senescence of leaves and haulms [18].

#### 2.5.2 Growth parameters

The heights of ten randomly taken plants grown in the net plot area were measured from the level of ground surface to the tip of the main stem using ruler at 50% flowering and the mean values were computed for further analysis. Similarly, stem number per hill was recorded by counting the main stems of ten randomly selected hills in the net plot area at 50% flowering. Only stems arising from the mother tuber were considered as main stem.

#### 2.5.3 Yield parameters

Tubers which were harvested from the net plot were categorized as very small (<25 g), small (25–38 g), medium (39–75 g), and large (>75 g) based on the size category described by Lung’aho et al. [16]. Each category was weighed separately and converted to t ha^−1^. Tubers that are free of mechanical, disease and insect pest damages and greater than or equal to 25 g were considered as marketable [19]. The weight of such tubers obtained from the net plots was measured in kilogram using scaled balance and converted to t ha^−1^. On the other hand, tubers that are damaged, misshaped, decayed and less than 25 g were considered as unmarketable [19].The weights of such tubers obtained from each net plot were measured in kilogram using scaled balance and converted to t ha^−1^. Summation of marketable and unmarketable yields resulted total tuber yield.

### 2.6 Data analysis

The collected data of all parameters of potato were subjected to two-way Statistical Analysis of Variance (ANOVA) using Statistical Analysis Software [20] version 9.2. Whenever treatment effects were significant, mean separations were conducted using Least Significant Difference (LSD) depending on ANOVA results [21].

### 2.7 Economic analysis

The analysis of partial budget and marginal rate of return was done using the procedures described by CIMMYT [22]. The costs of seed tubers were considered as a variable cost to calculate marginal rate of analysis. The average labor and fertilizer costs were also constant for all treatments. Marginal rate of return was calculated as a change of net benefit divided by change of cost in the treatment [22].

The article "Growth and tuber yield responses of potato (Solanum tuberosum L.) varieties to seed tuber size in northwest highlands of Ethiopia" was retracted in 2025. Reason: plagiarism.

## 3 Results and discussion

### 3.1 Phenological parameters of potato

#### 3.1.1 Days to 50% emergence

Variety (P < 0.001) and tuber size (P < 0.01) influenced days to 50% plant emergence of potato plants. Their interaction effect (P > 0.05) however did not affect days to 50% emergence of potato. Local variety (*Key Dinch*) emerged earlier (13.56 days) compared to the three improved varieties used in the present study (Table 1). Gudanie variety took longer days to emerge (19.78 days) followed by Shonkolla and Belete. Variation between varieties in terms of emergence could be attributed to the genetic difference among varieties. Differences in days to emergence among potato varieties, which was associated with the genetic makeup, were also observed by Dash et al. [23] and Fentaw et al. [24].

**Table 1:** Phenological parameters of potato plants influenced by variety and seed tuber size.

Treatment		
(a) Variety	Days to 50% emergence	Days to 50% flowering
Belete	16.67^b^	65.67^b^
Shonkolla	16.78^b^	66.44^b^
Gudanie	19.78^a^	69.22^a^
Local	13.56^c^	56.78^c^
Sign	***	***
LSD (p = 0.05)	1.28	1.08
(b) Seed tuber size category		
Small (31.5 ± 2.5 g)	17.92^a^	65.42^a^
Medium (57 ± 2.5 g)	16.50^b^	64.33^b^
Large (77.5 ± 2.5 g)	15.67^b^	63.83^b^
Sign	**	**
LSD (0.05)	1.11	0.931
CV (%)	7.85	1.70

*** = very highly significant at P < 0.001; ** = highly significant at P < 0.01; means followed by the same letter(s) within a column are not significantly different at p < 0.05; CV = coefficient of variation; LSD = Least Significant Difference.

Large-sized tubers emerged earlier (15.67 days) compared to the small-sized tubers (17.92 days) as indicated in Table 1. There was a general trend of increasing days to emergence with decreased seed tuber size. This might be due to the fact that large tubers have sufficiently more stored reserve foods that provide an optimal supply of carbohydrate for emergence than the small-sized seed tubers. Rojoni et al. [25] and Ebrahim et al. [14] also reported early germination and emergence of large seed classes because of the availability of more food materials while smaller seed classes emerged relatively late.

#### 3.1.2 Days to 50% flowering

Days to flowering was very highly significantly (P < 0.001) and highly significant (P < 0.01) influenced by the main effect of variety and tuber size, respectively. However, the interaction effects of both factors had not influenced this parameter. The results indicate that local variety flowered significantly earlier (56.78 days) as compared to the improved varieties tested. Gudanie variety took longer time (69.22 days) to reach 50% flowering (Table 1). The observed variation in terms of days to 50% flowering could be attributed to intrinsic or genetic variation of the varieties in completing their vegetative growth and variation in environmental adaptability among the varieties. Similar study confirmed early flowering of local variety compared to the improved varieties [18,26].

The article "Growth and tuber yield responses of potato (Solanum tuberosum L.) varieties to seed tuber size in northwest highlands of Ethiopia" was retracted in 2025. Reason: plagiarism.

Plants from small-sized tubers required more days to reach 50% flowering (65.42 days) whereas potato plants from large-sized tubers flowered early (63.83 days) (Table 1). The variation in 50% flowering of plants raised from small-sized seed tubers might be due to longer emergence days that also extended days to 50% flowering than large-sized seed tubers. Plants from small-sized seed tubers required significantly more days to reach 50% flowering than those from large-sized seed tubers [14]. Early flowering of potato plants sourced from large-sized seed tubers was directly associated with their early emergence in the present study, which is similar with the findings of Masarirambi et al. [27].

#### 3.1.3 Days to 90% maturity

Variety and tuber size influenced (P < 0.001) days to maturity of potato plants while their interaction significantly (P < 0.05) influenced this parameter. Plants from large-sized seed tubers matured earlier while plants from small-sized seed tuber matured late. Local variety planted with large-sized seed tubers matured earlier (91.67 days) while Gudanie variety planted with small-sized seed tubers required more days to mature (Table 2). Studies also confirmed early maturity of plants grown from large-sized seed tubers than those grown from small sized seed tubers [14]. Early maturity observed in the present study is also related with early emergence and flowering. Potato plants, which emerged and flowered early, were also matured early.

**Table 2:** Interaction effect of variety and seed tuber size on maturity and plant height of potato.

Variety	Seed tuber size category	Day to 90% maturity (days)	Plant height (cm)
Belete	Small	108.00^cd^	44.17ef
	Medium	105.33^e^	47.47de
	Large	101.67^f^	49.37cd
Shonkolla	Small	109.33^c^	47.73de
	Medium	108.67^cd^	49.13cd
	Large	106.67^de^	52.73bc
Gudanie	Small	123.00^a^	51.47bcd
	Medium	121.33^ab^	55.73b
	Large	119.67^b^	65.13a
Local	Small	100.33^fg^	33.50g
	Medium	98.00^g^	41.53f
	Large	91.67^h^	47.0de
Sign		*	*
LSD (0.05)		2.66	4.58
CV (%)		1.46	5.55

* = significant at P < 0.05; means followed by the same letter (s) in column are not significantly different at p < 0.05; CV = coefficient of variation; LSD = Least Significant Difference.

The article "Growth and tuber yield responses of potato (Solanum tuberosum L.) varieties to seed tuber size in northwest highlands of Ethiopia" was retracted in 2025. Reason: plagiarism.

Vegetation period for potato varieties varied from 90 to 124 days [28], which is in harmony with the results of the present study. Time required to reach maturity is a varietal characteristic which of course can be influenced by planting date, climatic condition and adopted cultivation practices [18,29].

### 3.2 Growth parameters of potato as influenced by variety and seed tuber size

#### 3.2.1 Plant height

Variety and seed tuber size as well as their interaction influenced plant heights of potatoes. Large-sized seed tubers of Gudanie variety produced the longest plants (65.13 cm) while small-sized seed tubers of the local variety produced the shortest plants (33.50 cm) as indicated in Table 2. The difference in plant height could be attributed to genetic variations among the varieties. Gudanie variety also recorded the tallest plants in the results of other scholars [29,30].

Plant heights of potato were increased as the seed tuber size increased from small to large, which is obviously associated with the more food reserves stored in large-sized tubers compared to small and medium-sized tubers. Increased plant height with increasing seed tuber size was also reported by different researchers [25,31]. In consistent to the present study, tallest potato plants were produced from larger-sized tubers of Gudanie variety whereas the shortest plants were recorded from small-sized tubers of the local variety [14].

#### 3.2.2 Stem number

Stem number of potato is the most important parameter that contributes for yielding potential of potato. It was very highly significantly (P < 0.001) influenced by variety and seed tuber size. However, the interaction of the two factors did not influence this parameter significantly. Gudanie variety produced the highest number of stem per hill (6.51) while Belete variety produced the least stem numbers (Table 3), which could be attributed with the inherent genetic variation in the number of eyes on tubers. Genetic differences among potato varieties influence the number of sprouts or eyes on tubers, which in turn influence the main stem numbers [26]. Stem numbers sourced from a given tuber vary considerably with variety, storage condition, tuber size, number of viable sprouts at planting, sprout damage at the time of planting, physiological age of the seed tuber and growth conditions [32]. According to Ebrahim et al. [14] Gudanie variety produced highest stem number per hill compared to local and Belete varieties.

The article "Growth and tuber yield responses of potato (Solanum tuberosum L.) varieties to seed tuber size in northwest highlands of Ethiopia" was retracted in 2025. Reason: plagiarism.

**Table 3:** Stem number responses of potato as influenced by the main effects of variety and seed tuber size.

Treatment	
(a) Variety	Stem number (count hill^−1^)
Belete	4.86c
Shonkolla	6.31a
Gudanie	6.51a
Local	5.90b
Sign	***
LSD (0.05)	0.40
(b) Seed tuber size category	
Small (31.5 ± 2.5 g)	4.73b
Medium (57 ± 2.5 g)	6.31a
Large (77.5 ± 2.5 g)	6.65a
Sign	***
LSD (0.05)	0.35
CV (%)	6.95

*** = very highly significant at P < 0.001; means followed by the same letter (s) within a column are not significantly different at P < 0.05; CV = coefficient of variation; LSD = Least Significant Difference.

In terms of tuber size, highest number of main stems per hill (6.65) was recorded from large-sized tubers while the least number of potato stems (4.73) was observed from small-sized tubers (Table 3). The results clearly indicated that increasing the seed tuber size increased the number of main stems in both varieties. Large-sized seed tubers generally have relatively many eyes, which consequently could produce more main stems per hill. Varying number of stems based on differences in seed tuber size was also reported by other researchers, where larger tubers produced more sprouts and consequently more stems per plant compared to smaller seed tubers [27,31].

### 3.3 Yield and yield related parameters

#### 3.3.1 Very small-sized (<25 g) tuber yield

Variety and seed tuber size of potato affected (P < 0.001) very small-sized tuber yield while the combination of the two factors did not influence this parameter. Local variety produced the highest very small-sized tuber yield (1.65 t ha^−1^), which was at par with that of Shonkolla variety. On the other hand, the lowest very small-sized tubers yield (0.91 t ha^−1^) was obtained from Belete variety, which was statistically similar with the yield of Gudanie variety (Fig. 1a). The difference in very small-sized tuber yield could be associated with the inherent characteristics of potato varieties. According to Binalfew et al. [33] tuber size of potato is hereditary trait. The authors also reported that tuber size of Belete variety is naturally bigger compared to other varieties commonly produced in the Ethiopia, which is also observed in the present study. Very small-sized tubers have generally low market values.

**Fig. 1:** Influence of variety (a) and seed tuber size (b) on very small-sized tuber yield (t ha-1) of potato. Note: Mean values with the same letter within the group are statistically similar at p < 0.05.

The use of different seed tuber sizes as a planting material had a significant effect on very small-sized tuber yield. The highest yield of very small-sized tubers was obtained when smaller-sized seed tubers were used as planting materials. Using small-sized tubers as planting material increased very small-sized tuber yield by 39.36% and 56.38% compared to using medium-, and large-sized seed tubers, respectively (Fig. 1b). The fact that small-sized seed tubers have less number of eyes and minimum stored foods; it reduces the vegetative growth and consequently produces very small-sized potato tubers. Similar results also showed that plants sourced from small-sized seed tubers produced low number of eyes and reduced vegetative growth [31].

The article "Growth and tuber yield responses of potato (Solanum tuberosum L.) varieties to seed tuber size in northwest highlands of Ethiopia" was retracted in 2025. Reason: plagiarism.

#### 3.3.2 Small-sized (25–38 g) tuber yield

Variety and seed tuber size influenced (P < 0.001) the small-sized tuber yield of potatoes. Their interaction however did not influence the yield of small-sized tubers. Gudanie variety recorded the highest (5.89 t ha^−1^) small-sized tuber yield while local variety produced the lowest yield (2.88 t ha^−1^) (Fig. 2a). The difference in small-sized tuber yield observed between varieties in the present study is obviously due to the genetic makeup of the varieties. In this regard, Binalfew et al. [33] reported the heritability of grades of potato tubers.

**Fig. 2:** Influence of variety (a) and seed tuber size (b) on small-sized tuber yield (t ha^−1^) of potato. Note: Mean values with the same letter within the group are statistically similar at p < 0.05.

The small-sized tuber yield was also influenced by seed tuber size of potatoes where large-sized seed tubers recorded the highest small-sized tuber yield (4.98 t ha^−1^). Small-sized seed tubers on the other hand recorded the lowest yield (3.34 t ha^−1^) as indicated in Fig. 2b. Generally, as the seed tuber size increased the proportional yield of small-sized tubers also increased. This is probably associated with the production of high number of main stems per hill related to large-sized seed tubers that exerts high competition among potato plants and leads to the production of high small-sized tuber yield. Similar findings were also reported by Lung’aho et al. [16] where big seed tubers produced more main stems that compete for growth factors and lead to the production of small-sized potato tubers.

#### 3.3.3 Medium-sized (39–75 g) tuber yield

Seed tuber size and variety influenced (P < 0.001) the medium-sized tuber yield of potato. However, the two factors did not interact to influence this parameter of potato. Gudanie variety produced significantly highest medium-sized tuber yield (11.04 t ha^−1^) while local variety the lowest yield (6.16 t ha^−1^) as indicated in Fig. 3a. The results clearly showed that medium-sized tuber yields vary with the genetic makeup of potato varieties, which is in line with the findings of Sharma et al. [34].

The article "Growth and tuber yield responses of potato (Solanum tuberosum L.) varieties to seed tuber size in northwest highlands of Ethiopia" was retracted in 2025. Reason: plagiarism.

**Fig. 3:** Influence of variety (a) and seed tuber size (b) on medium-sized tuber yield (t ha^−1^) of potato. Note: Mean values with the same letter within the group are statistically similar at p < 0.05.

The yield of medium-sized tuber yield in potato was also affected by seed tuber size of potatoes. Large-sized seed tubers produced significantly highest medium-sized tuber yield (10.50 t ha^−1^) whereas small-sized seed tubers produced the lowest medium-sized tuber yield (7.25 t ha^−1^) (Fig. 3b). Medium-sized tuber yield of potato was generally increased as the seed tuber size increased from small to large, which could be associated with the production of optimum number of main stems that in turn produces high medium-sized tuber yield. Using large-sized seed tubers also produced the highest medium-sized tuber yield as reported by Dagne et al. [31].

#### 3.3.4 Large-sized (>75 g) tuber yield

Variety and seed tuber size in their main effects (P < 0.001) and their interaction effects (P < 0.05) influenced the large-sized tuber yield of potatoes. Large-sized seed tubers combined with Belete variety produced the highest large-sized tuber yield (25.76 t ha^−1^) while the lowest large-sized tuber yield (5.28 t ha^−1^) was recorded by the combination of local variety and small-sized seed tuber as indicated in Fig. 4. Tuber size of potatoes is influenced by agronomic practices and genetic makeup of the varieties [35]. Genetically Belete variety is producing relatively big tubers [34]. It is also observed in the present study. According to Dagne et al. [31] 2018) big seed tubers have relatively high food reserves that could have significant effect on growth and development of plants and consequently enhance large-sized tuber yield of potato.

**Fig. 4:** Interaction effect of variety and seed tuber size on large-sized tuber yield of potato. Note: Mean values with the same letter/s are statistically similar at P < 0.05.

#### 3.3.5 Total tuber yield

The analysis of variance showed that variety and seed tuber size in their main (P < 0.001) effects as well as their interaction (P < 0.05) effects influenced total tuber yield of potato. Highest total tuber yield was obtained when Belete (39.97 t ha^−1^) and Gudanie (39.85 t ha^−1^) varieties were planted using large-sized seed tubers whereas the lowest marketable tuber yield (15.00 t ha^−1^) was obtained from small-sized seed tubers of local variety (Table 4).

**Table 4:** Interaction effect of variety and seed tuber size on tuber yield of potato.

Variety	Seed tuber size category (g)	Total tuber yield (t ha^−1^)	Marketable tuber yield (t ha^−1^)
Belete	Small	31.27cd	28.74de
	Medium	32.33bc	31.10cd
	Large	39.97a	39.13a
Shonkolla	Small	27.29de	24.64ef
	Medium	32.47ab	29.47d
	Large	31.25cd	31.12cd
Gudanie	Small	26.36e	23.79f
	Medium	35.76ab	34.32bc
	Large	39.85a	38.63ab
Local	Small	15.00g	12.12h
	Medium	17.61fg	15.01gh
	Large	20.86f	18.94g
Sign		*	*
LSD (0.05)		4.4.7	4.32
CV (%)		9.04	9.35

* = significant at P < 0.05; means followed by the same letter (s) are not significantly different at p < 0.05; CV = coefficient of variation; LSD = Least Significant Difference.

The article "Growth and tuber yield responses of potato (Solanum tuberosum L.) varieties to seed tuber size in northwest highlands of Ethiopia" was retracted in 2025. Reason: plagiarism.

Potato varieties differ in their yielding capacities, which is associated with their genetic makeup [ [14,23,24,26,36,37]]. According to the researchers, improved varieties have generally high yielding capacities compared to the landrace varieties, which is in line with the findings of the present study. The results of the present study clearly showed that total tuber yield of potato was increased as the seed tuber size increased from small to large. The presence of numerous eyes on large-sized tubers lead to the production of several stems that produce more tubers and consequently higher total tuber yield as indicated in the present study. Increasing the total tuber yield of potato by increasing the seed tuber size was also reported by other researches [25,31].

#### 3.3.6 Marketable tuber yield

Marketable tuber yield is the most important parameters of potato, which influence the economics of potato production. Variety and seed tuber size in their main (P < 0.001) effects as well as in their interaction effect (P < 0.05) influenced the marketable tuber yield. Belete and Gudanie varieties produced more marketable tuber yield compared to Shonkolla variety of potato while local variety produced the lowest marketable yield. Similarly, the use of large-sized seed tubers recorded more marketable yield compared to other seed categories. The treatment combination of Belete variety and large-sized seed tuber recorded the highest marketable tuber yield (39.13 t ha^−1^), which was however statistically similar with the yield obtained from the treatment combination of Gudanie variety and large-sized seed tuber. Local variety combined with small-sized seed tuber produced the lowest marketable tuber yield (Table 4). In the present study improved potato varieties generally produced more marketable yield compared to the local variety, which was also reported by other scholars [14,23,26].

The increased marketable tuber yield with increased seed tuber size observed in the present study is probably associated with the presence of relatively more buds and food reserves, which enhance sprouting and vegetative growth. Moreover, improved photosynthetic activities and accumulation of assimilate lead to the production of more marketable tuber yield [25]. Marketable tuber yield was also increased when the seed tuber size increased from small to large seed tuber sizes [14].

The article "Growth and tuber yield responses of potato (Solanum tuberosum L.) varieties to seed tuber size in northwest highlands of Ethiopia" was retracted in 2025. Reason: plagiarism.

#### 3.3.7 Unmarketable tuber yield

Variety and seed tuber size influenced (P < 0.001) unmarketable tuber yield of potatoes. However, the interaction of the two factors did not influence the unmarketable tuber yield. Generally improved varieties produced relatively low unmarketable yield compared to the local variety (2.47 t ha^−1^). On the other hand, potato plants grown from small-sized seed tubers recorded the highest unmarketable tuber yield, while plants from large-sized seed tubers the lowest unmarketable tuber yield (results not included).

The observed high unmarketable tuber yield of local variety might be associated with the genetic makeup of the variety [30]. In this regard, Getie et al. [26] reported that local (*Key Dinch)* variety produced highest unmarketable tuber yield than the improved potato varieties.

The decrease in unmarketable tuber yield by increased seed tuber size recorded in the present study is obviously associated with the presence of high reserve foods in large-sized tubers that facilitate the vegetative growth and tuber development, which in turn reduce the yield of very small-sized tubers (unmarketable yield) as indicated in the present study. Similar results were also reported by Ebrahim et al. [14] where large-sized seed tubers produced relatively low unmarketable tuber yield of potato.

### 3.4 Partial budget analysis of potato as influenced by variety and seed tuber size

Partial budget analysis considers total variable costs and net benefits of each treatment. In the present study, marketable yield was downscaled by 10% to make it comparable to farmer′s production conditions. The field sale price of potato at the time of harvesting was 5.00 ETB per kg. According to the partial budget analysis described by CIMMYT [22] Gudanie variety planted with large-sized seed tubers recorded the highest net benefit (131,376.50 ETB ha^−1^) followed by the combination of Belete variety and large-sized seed tubers while the combination of small-sized seed tuber and local variety recorded the lowest net benefit (Table 5).

**Table 5:** Partial budget of potato influenced by variety and seed tuber size.

Variety	Seed tuber size category	Seed cost (ETB ha^−1^)	Marketable Yield (t ha^−1^)	AdY (t ha^−1^)	Gross income (ETB ha^−1^)	Net benefit (ETB ha^−1^)
Belete	Small	18480.00	28.74	25.87	129330.00	110850.00
	Medium	33435.60	31.10	27.99	139950.00	106514.40
	large	45751.20	39.13	35.22	176085.00	130333.80
Shonkolla	Small	17430.00	24.64	22.18	110880.00	93450.00
	Medium	31535.90	29.47	26.52	132615.00	101079.20
	large	43151.70	31.12	28.01	140040.00	96888.30
Gudanie	Small	17150.00	23.79	21.41	107055.00	89905.00
	Medium	31029.30	34.32	30.89	154440.00	123410.80
	large	42458.50	38.63	34.77	173835.00	131376.50
Local	Small	9730.00	12.12	10.91	54540.00	44810.00
	Medium	17604.40	15.01	13.51	67545.00	49940.70
	large	24088.70	18.94	17.05	85230.00	61141.30

Seed tuber costs for Belete, Shonkolla, Gudanie and local varieties were 13.20, 12.45, 12.25 and 6.95 ETB kg^−1^, respectively; Sale price of potato at farm gate was 5.0 ETB kg^−1^ for all varieties; AdY = Adjusted marketable Yield.

The article "Growth and tuber yield responses of potato (Solanum tuberosum L.) varieties to seed tuber size in northwest highlands of Ethiopia" was retracted in 2025. Reason: plagiarism.

Small-sized seed tubers of Belete variety recorded the highest marginal rate of returns (1657.14%), but recorded relatively low net benefit (Table 6). Large-sized seed tuber combined with Gudanie and Belete varieties performed best in terms of net benefits (Table 5). The treatment combination of Belete variety and large-sized seed tuber was however dominated and discarded from MRR analysis (Table 6), which is obviously associated with the required high quantity of seed tubers that intern increases the seed cost (variable cost). According to CIMMYT [22], any treatment that had a net benefit less than (or equal to) those of a treatment with lower total variable costs is dominated and discarded from the MRR analysis. The combination of Gudanie variety with large-sized seed tuber on the other hand recorded a marginal rate of return less than 100% (69.7%), which is unacceptable in the case of developing countries like Ethiopia.

**Table 6:** Marginal rate of return of potato as influenced by variety and seed tuber size.

Treatment combinations	Total variable cost (ETB ha^−1^)	Net benefit (ETB ha^−1^)	Dominance Analysis	MRR (%)
Local × Small	9730.00	44810.00		–
Gudanie × Small	17150.00	89905.00		607.75
Shonkolla × Small	17430.00	93450.00		1266.07
Local × Medium	17604.35	49945.65	DO	
Belete × Small	18480.00	110850.00		1657.14
Local × Large	24088.70	61141.30	DO	
Gudanie × Medium	31029.25	123410.75		100.09
Shonkolla × Medium	31535.85	101079.15	DO	
Belete × Medium	33435.60	106514.40	DO	
Gudanie × Large	42458.50	131376.50		69.70
Shonkolla x Large	43151.70	96888.30	DO	
Belete × Large	45751.20	130333.80	DO	

Notes: DO = Dominated; MRR = marginal rate of return.

## 4 Conclusion and recommendation

The results of the present study clearly showed that variety and seed tuber size influenced almost all the tested phenological, growth, and yield parameters of potato. The improved varieties generally performed well in all the tested parameters of potato compared to the local variety. Increasing the seed tuber size from small (31.5 ± 2.5 g) to large (77.5 ± 2.5 g) increased the tuber yield of potato. Belete (39.13 t ha^−1^) and Gudanie (38.63 t ha^−1^) varieties each combined with large-sized seed tubers produced the highest marketable tuber yields. The same treatment combinations also recorded highest net benefits. Generally, using large-sized seed tubers as planting materials leads either to domination of the treatment combinations (Belete, Shonkolla and local) or results unacceptable MRR in the case of Gudanie variety (<100%). On the other hand, small-sized seed tubers result relatively higher MRRs, but relatively low net benefit. Optimization of seed tuber size is therefore necessary to increase productivity and profitability of potato. Accordingly, Gudanie variety combined with medium-sized seed tuber (57 ± 2.5 g) recorded relatively higher net benefit (123,410.80 ETB ha^−1^) with acceptable MRR (100.9%). This treatment combination could be therefore recommended for economical production of potato and improvement of the income and food security of smallholder farmers in the study area and areas with similar agro-ecologies.

The article "Growth and tuber yield responses of potato (Solanum tuberosum L.) varieties to seed tuber size in northwest highlands of Ethiopia" was retracted in 2025. Reason: plagiarism.

## Author contribution statement

Daniel Asnake: Conceived and designed the experiments; Performed the experiments.

Melkamu Alemayehu: Conceived and designed the experiments; Wrote the paper.

Semagn Asredie: Analyzed and interpreted the data; Contributed reagents, materials, analysis tools or data.

## Funding statement

This research did not receive any specific grant from funding agencies in the public, commercial, or not-for-profit sectors.

## Data availability statement

Data will be made available on request.

## Declaration of interest’s statement

The authors declare no competing interests.

## Additional information

No additional information is available for this paper.
